# Equalized Grey Wolf Optimizer with Refraction Opposite Learning

**DOI:** 10.1155/2022/2721490

**Published:** 2022-05-11

**Authors:** Lijun Sun, Binbin Feng, Tianfei Chen, Dongliang Zhao, Yan Xin

**Affiliations:** ^1^Key Laboratory of Grain Information Processing and Control, Ministry of Education, Henan University of Technology, Zhengzhou 450001, China; ^2^Zhengzhou Key Laboratory of Machine Perception and Intelligent System, Henan University of Technology, Zhengzhou 450001, China; ^3^College of Information Science and Engineering, Henan University of Technology, Zhengzhou 450001, China

## Abstract

Grey wolf optimizer (GWO) is a global search algorithm based on grey wolf hunting activity. However, the traditional GWO is prone to fall into local optimum, affecting the performance of the algorithm. Therefore, to solve this problem, an equalized grey wolf optimizer with refraction opposite learning (REGWO) is proposed in this study. In REGWO, the issue about the low swarm population variety of GWO in the late iteration is well overcome by the opposing learning of refraction. In addition, the equilibrium pool strategy reduces the likelihood of wolves going to the local extremum. To investigate the effectiveness of REGWO, it is evaluated on 21 widely used benchmark functions and IEEE CEC 2019 test functions. Experimental results show/ that REGWO performs better than the other competitors on most benchmarks.

## 1. Introduction

Complex optimization problems in practice are often discontinuous, nondifferentiable, and nonconvex. Prior to the advent of metaheuristic optimization technology [1], the most widely used optimization methods were the gradient descent algorithm and the Gauss-Newton method [2]. However, the gradient-based optimization approach is prone to obtaining the local extremum interference, resulting in a reduction in optimization precision. On the contrary, metaheuristic optimization algorithms are able to identify optimum or near-optimum solutions within an acceptable time. Therefore, many scholars have researched metaheuristic optimization algorithms in order to address challenging optimization problems, such as particle swarm algorithm (PSO) [3], artificial bee colony algorithm (ABC) [4], ant colony optimization algorithm (ACO) [5], slime mould algorithm (SMA) [6], hunger games search (HGS) [7], Runge–Kutta method (RUN) [8], grey wolf optimizer (GWO) [9], weighted mean of vectors (INFO) [10], and so on. Among these algorithms, GWO has become the focus of research in recent years due to its advantages, such as few parameters and straightforward principle.

GWO is a swarm intelligence stochastic optimization algorithm introduced in 2014, as a result of information interaction between the social level and hunting behavior of grey wolves in nature [9]. GWO is an effective metaheuristic, and it attracted the interest of academics when it was initially introduced. It has been widely used in many fields such as feature selection [11, 12], image processing [13, 14], path planning [15], weld shop inverse scheduling [16], and so on. In GWO, the search process is guided by the leading wolves in each iteration, which shows great convergence toward leading wolves. The leading wolves sometimes fall into the local extremum, especially in multimodal problems. However, when leading wolves get trapped at local optima, other individuals in the population are also vulnerable to local extremes. This is the cause of the decrease in population diversity. Therefore, the standard GWO suffers from the same issues as most swarm intelligence algorithms, such as lack of the population diversity and ease of falling into local optimum [17].

The motivation of this paper is to solve the above problem; in order to overcome these weaknesses, an equalized grey wolf optimizer with refraction opposite learning (REGWO) is proposed in this paper. In REGWO, two search strategies with different features are introduced to generate candidate solutions. Among them, the opposite learning of refraction strategy is inspired by the principle of light refraction in nature. This strategy is introduced to improve population diversity during the search and expand the scope of solution space. At the same time, the fuzzy theory is used to adjust the parameter so that the refraction solution is more random and the algorithm can find more potential solutions. Moreover, the equilibrium pool strategy is designed to impair the leadership of the leading wolves. This method can make wolves update their position following nonoptimal solution with a certain probability, so wolves have the ability to jump out of the local extremum even when the optimal solution falls into the local optimum. REGWO can achieve better performance by combining the aforementioned tactics.

The remainder of this paper is organized as follows. The related work is discussed in Section 2.  Section 3 presents the original GWO algorithm. The proposed REGWO algorithm is introduced in Section 4. In Section 5, the performance of the proposed REGWO is evaluated on different benchmark functions; furthermore, the significance of the results is proved by statistical analysis. Finally, we end the paper with conclusions and future work in Section 6.

## 2. Related Work

The metaheuristic optimization algorithms have been widely used to solve optimization problems. These algorithms are divided into three categories: physics-based algorithms, evolutionary algorithms, and swarm intelligence algorithms. Physics-based algorithms mimic the physical rules in nature in which the individuals communicate around the search space by the physical concepts, such as inertia force, light refraction law, gravitational force, and so on. There are some popular algorithms in this category, such as atom search optimization (ASO) [18] and Henry gas solubility optimization [19]. Evolutionary algorithms are a kind of iterative optimization algorithms simulating natural evolutionary processes. The best individuals are combined to form a new generation, which is the main advantage of EAs because it promotes population improvement during iteration, such as genetic algorithm (GA) [20] and differential evolution (DE) [21]. Swarm intelligence algorithms are inspired by the collective behavior of swarm organisms, such as bird flocking, animal grazing, and so on. Individuals in a population with cooperation and interaction move collectively to the promising areas in the search space. Some recently proposed swarm-based intelligence algorithms are grey wolf optimizer (GWO) [9], monarch butterfly optimization (MBO) [22], moth search algorithm (MSA) [23], Harris hawks optimization (HHO) [24], colony predation algorithm (CPA) [25], and so on.

Swarm intelligence algorithms have been shown to be effective at solving optimization problems, but they may fall into local optimum and loss of diversity. As a result, some scholars have proposed modified variations to tackle the flaws. DEWCO algorithm has improved the initial population through a hyperheuristic to increase its convergence speed [26]. EFSABC algorithm is proposed by a search strategy for group escape and foraging based on Levy flight to exit from local optima [27].

GWO is a kind of swarm intelligence algorithm, which imitates the social level of wolves and the group hunting behavior. It has fewer parameters and is easy to implement. Therefore, this algorithm has been widely used to solve different optimization problems, such as multidimensional knapsack problem [28], path planning [29], parameter estimation [30], economic dispatch [31], feature selection [32], large scale unit commitment problem [33], wind speed forecasting [34], and so on.

In recent years, numerous scholars have developed variants of the basic GWO to address the weaknesses of GWO and provide better performance. Three different position update methods are proposed [35], which are weighted average, fitness-based, and fuzzy logic. Further experimental analysis reveals that the GWO improved using the fuzzy logic method has better performance. In order to improve the search ability of grey wolf, a modified algorithm RW-GWO based on a random walk has been imported [36]. A cellular grey wolf optimizer with a topological structure (CGWO) is introduced. In CGWO, each wolf has its own topological neighbors, and interactions among wolves are restricted to their neighbors, which favors exploitation. Furthermore, the information diffusion mechanism by overlap among neighbors can allow maintaining the population diversity for longer, usually contributing to exploration [37]. Grey wolf optimizer with crossover and opposition-based learning (GWO-XOBL) is presented to the jump out local optima [38]. An improved grey wolf optimizer is proposed using the explorative equation and opposition-based learning (OBL) [39]. To get a more stable sense of balance between exploitation and exploration, a new modified GWO called memory-based grey wolf optimizer (mGWO) is introduced [40]. Randomized balanced grey wolf optimizer (RBGWO), which improves the overall efficiency of the search process by establishing a balance between its exploitation and exploration capability incorporating three successive enhancement strategies equipped with a social hierarchy mechanism and random walk with student's t-distributed random numbers [41]. By dividing the search process into three stages and using different population updating strategies at each stage, an improved GWO called multistage grey wolf optimizer (MGWO) is proposed; the MGWO is improved while maintaining a certain convergence speed [42].

Another area of interest for researchers is to combine other evolutionary algorithms or operators to improve the performance of GWO. PSO-GWO algorithm merged with PSO [43], the idea of PSO was introduced into the GWO to update the position information of each individual using the optimal value of the individual and the optimal value of the group, which enhanced the diversity of the population and improved the global search ability. The crossover operator is introduced into GWO to promote population diversity [44]. The purpose of the crossover operator is to enhance information sharing among individuals in the population. At the same time, the search accuracy and convergence speed of the algorithm are improved. Grey wolf optimizer has been hybridized with differential evolution (DE) mutation, and two versions, namely DE-GWO and gDE-GWO, have been proposed to avoid the stagnation of the solution [45]. To improve the performance of the GWO, a new variant of the GWO called a mutation-driven modified grey wolf optimizer and denoted by MDM-GWO is proposed. The MDM-GWO combines a new update search mechanism, modified control parameter, mutation-driven scheme, and greedy approach of selection in the search procedure of the GWO [46]. SCGWO algorithm combines GWO with an improved spread strategy and a chaotic local search mechanism to accelerate the convergence rate of the evolving agents [47]. GWO variant enhanced with a covariance matrix adaptation evolution strategy, Levy fight mechanism, and orthogonal learning strategy named GWOCMALOL is proposed. GWOCMALOL algorithm uses these strategies to bring more effective exploratory inclinations [48].

According to the various improvement strategies mentioned above, the main aim of the GWO variants is to improve search accuracy and convergence speed. Although the above GWOs can overcome some drawbacks of the original GWO, GWO still faces the problem of poor global exploration ability in the late iteration. Therefore, an equalized grey wolf optimizer with refraction opposite learning (REGWO) is presented in this paper.

## 3. Grey Wolf Optimizer

GWO is a typical swarm intelligence optimization algorithm. The model of GWO originates from the leading class and hunting behavior of grey wolves. There is a clear division of labor and cooperation among grey wolf individuals. As shown in Figure 1, the grey wolf population is separated into four levels, namely *α*, *β, δ*, and *ω* wolves. The first layer is the *α* wolf, and the next layer is called the *β* wolf. The *δ* wolf is located in the third layer. The grey wolf in the population is called the *ω* wolf (search wolf), which is located in the bottom layer. The *α*, *β*, and *δ* wolves are called leading wolves, and their number is set to 1. In GWO, the *ω* wolf must update its position to obtain the optimal solution, and *α*, *β*, and *δ* wolves represent the optimal value, suboptimal value, and third optimal value, respectively. The hunting process of grey wolves is mainly guided by *α*, *β*, and *δ* wolves, and *ω* wolves update iteratively according to the position of leading wolves.

The formula of the grey wolf around prey can be expressed as follows [41]:

(1) $$\begin{array}{c} D=C\circ X_{p}\left(t\right)-X\left(t\right),\\ X\left(t+1\right)=X_{p}\left(t\right)-A\circ D. \end{array}$$

Here, *t* is the current number of iterations; ∘ is the Hadamard product operation; ***X***_*p*_ and ***X*** denote the position vector of the prey and a grey wolf, respectively; and the calculation formulas of random vectors ***A*** and ***C*** are as follows:

(2) $$\begin{array}{c} A=2a\circ r_{1}-a,\\ C=2r_{2}, \end{array}$$

where ***r***_1_ and ***r***_2_ are random vectors between [0, 1] and the vector ***a*** is linearly decreased from 2 to 0 over the course of iterations.

To better understand the optimization rules of GWO, the possible areas are shown in Figure 2 when the position of the grey wolf is updated. It can be seen from Figure 2 that *ω* wolf can reach different positions around the prey by adjusting the values of parameters ***A*** and ***C***. Furthermore, random variables *r*_1_ and *r*_2_ can assist search wolves to reach any of the points depicted in Figure 2. Parameters ***A*** and ***C*** are responsible for exploration and exploitation behavior in GWO. **A** is a random value between [−***a***, ***a***]. When ***A*** > 1 and ***C*** > 1, the population is inclined to exploration. In addition, when **A** < 1 and ***C*** < 1, the population is prone to exploitation.

The formulas of grey wolf tracking target prey are as follows [41]:

(3) $$\begin{array}{c} \left\{\begin{array}{c} D_{a}=C_{1}\circ X_{\alpha }-X,\\ D_{\beta }=C_{2}\circ X_{\beta }-X,\\ D_{\delta }=C_{3}\circ X_{\delta }-X, \end{array}\right.\\ \left\{\begin{array}{c} X_{1}=X_{\alpha }-A_{1}\circ D_{\alpha },\\ X_{2}=X_{\beta }-A_{2}\circ D_{\beta },\\ X_{3}=X_{\delta }-A_{3}\circ D_{\delta }, \end{array}\right.\\ X\left(t+1\right)=\frac{X_{1}+X_{2}+X_{3}}{3}. \end{array}$$

Here, ***D***_*α*_, ***D***_*β*_, and ***D***_*δ*_ denote the distance between *α*, *β*, and *δ* wolves and other individuals, respectively; ***X***_*α*_, ***X***_*β*_, and ***X***_*δ*_ represent the positions of *α*, *β*, and *δ*, severally, respectively; ***C***_1_, ***C***_2_, and ***C***_3_ are random vectors; ***X***_1_, ***X***_2_, and ***X***_3_ represent the step length and direction of *ω* wolf toward *α*, *β*, and *δ*, respectively; and *ω* wolf determines the final position according to equation (3).

## 4. Proposed Algorithm REGWO

To improve the global search ability of GWO, the opposite learning of refraction and equilibrium pool technique are introduced in this work. Opposite learning of refraction is chosen in the proposed algorithm to generate more potential solutions. Besides, the equilibrium pool strategy can achieve a better exploration by weakening the leadership of the leading wolf. The two strategies are introduced in Sections 4.1 and 4.2, respectively. The proposed algorithm is named REGWO and described in Section 4.3.

### 4.1. Opposite Learning of Refraction

The opposition-based learning (OBL) technique is proposed in 2005 [49]. The fundamental idea is to expand the search space of the population by calculating the opposite solution of the current solution, so as to select the candidate solution that is more suitable for the optimization problem. Applying this method to the optimization algorithm can effectively improve the search accuracy of the algorithm [50]. However, the standard OBL has certain shortcomings. OBL only speeds up the convergence of GWO and obtains only one opposite solution of fixed position. Therefore, the opposite solution may fall near the local optimal solution, causing the algorithm to fall into the local optimum with the iteration [51]. In order to tackle this problem, this paper introduces the refraction principle to improve the traditional opposite learning process. Refracted opposition-based learning (ROBL) strategy is based on the OBL, combined with the principle of light refraction to identify a better solution. ROBL strategy not only considers the opposite direction of individuals but also considers other directions of individuals. The schematic is shown in Figure 3.

In the one-dimensional space where the individual of the population is located, the *x*-axis is separated into the upper and lower parts. Above the *x*-axis is the natural vacuum part of the refraction model, and below the *x*-axis is the other propagation medium of the refraction model. In Figure 3, the search range of individuals on the *x*-axis is [*a*, *b*], that is, *x*∈[*a*, *b*], and the *y*-axis is normal. *x*′ is the incident point of the light source, and the length of the incident light segment *x*′*o* is denoted by *h*. The incident light refracts at the intersection *o*, and *x*′^*∗*^ is the refraction point; the length of refraction light segment *ox*′^*∗*^ is denoted by *h*^*∗*^; and *θ* and *φ* are the incidence angle and the refraction angle, respectively. The *x* coordinate (position) of intersection *o* is (*a* + *b*)/2, which is the midpoint of the individual search range [*a*, *b*]. From the geometric relationship in Figure 3, we can obtain

(4) $$\begin{array}{c} \sin\;\theta =\frac{\left(\left(a+b\right)/2-x\right)}{h}. \end{array}$$

(5) $$\begin{array}{c} \text{sin}\varphi =\frac{\left(x^{*}-\left(a+b\right)/2\right)}{h^{*}}. \end{array}$$

The refractive index (*n*=sin  *θ*/sin  *φ*) of light obtained by equations (4) and (5) is

(6) $$\begin{array}{c} n=\frac{\left(\left(\left(a+b\right)/2-x\right)/h\right)}{\left(\left(x^{*}-\left(a+b\right)/2\right)/h^{*}\right)}. \end{array}$$

Let *k* = *h*/*h*^*∗*^; equation (6) can be transformed into

(7) $$\begin{array}{c} \mathrm{kn}=\frac{\left(\left(a+b\right)/2-x\right)}{\left(x^{*}-\left(a+b\right)/2\right)}. \end{array}$$

According to equation (7), we can obtain

(8) $$\begin{array}{c} x^{*}=\frac{\left(a+b\right)/2-x}{kn}+\frac{a+b}{2}. \end{array}$$

When *n* and *k* are both 1, equation (8) is the standard opposite learning formula:

(9) $$\begin{array}{c} x^{*}=a+b-x. \end{array}$$

Obviously, the OBL strategy is a special case of the ROBL strategy. In order to improve the ability of GWO to jump out of the local extremum, the above ROBL model is applied to GWO. Since the individuals in GWO are multidimensional, equation (8) can be extended to the *D*-dimensional space as follows:

(10) $$\begin{array}{c} x_{i,j}^{*}=\frac{\left(a_{j}+b_{j}\right)/2-x_{i,j}}{kn}+\frac{a_{j}+b_{j}}{2}. \end{array}$$

Here, *x*_*i,j*_ represents the value of the *j*-th dimension of the *i*-th individual; *x*_*i*,*j*_^*∗*^ is the opposite solution obtained by the ROBL model; and *a*_*j*_ and *b*_*j*_ are the *j*-th dimension upper bound and lower bound, respectively.

As shown in Figure 3 and above, as the *k* value changes, the position of the opposite solution generated by (10) will be changed. That is to say, the adjustment of *k* improves the randomness of the solution. The *k* is calculated by

(11) $$\begin{array}{c} k\left(t\right)=k_{\max}-\frac{\left(k_{\max}-k_{\min}\right)t}{T}, \end{array}$$

where *k*_max_ = 1, *k*_min_ = 0, *t* denotes the current iteration number, and *T* is the total number of iterations.

Meanwhile, in order to make the decline rate of *k* well match the convergence rate of the fitness value, this paper proposes a method to adjust the *k* value as shown in Figure 4. The fuzzy membership degree *μ*_*k*_(*t*) of *k* is

(12) $$\begin{array}{c} \mu_{k}\left(t\right)=\frac{k\left(t\right)-k_{\min}}{k_{\max}-k_{\min}}, \end{array}$$

where *μ*_*k*_(*t*)∈[0,1], *μ*_*k*_(*t*) increases with the increase of *k*(*t*), *μ*_*k*_(*t*) decrease with the decrease of *k*(*t*), and the optimal fitness relative change rate *η* is

(13) $$\begin{array}{c} \eta =\frac{f\left(t\right)-f\left(t-10\right)}{f\left(t-10\right)}. \end{array}$$

Here, *f*(*t*)is the objective function, namely the optimal fitness value of the *t*-th iteration of the population; *f*(*t* − 10) represents the optimal fitness value of the (*t* − 10)-th iteration of the population; then *η* denotes the relative change rate of the optimal fitness value in 10 iterations of evolution; and when *η* value is large, it indicates that the change rate of the optimal fitness value is large, and at this time, the *k* value should be larger to improve global search capability; otherwise, when *η* value is small, it indicates that the change rate of the optimal fitness value is small, and at this time, the *k* value should be smaller. In the ROBL model, firstly, the current *η* and *μ*_*k*_(*t*) are judged. Then, the *k* of the next iteration is adaptively adjusted by fuzzy rules, which can accelerate the convergence speed of the algorithm.

Fuzzy rules to adjust (*k*):

 
*Rule 1.* If (*μ*_*k*_(*t*) > 0.5 and *η* > *γ*) or (*μ*_*k*_(*t*) ≤ 0.5 and *η* ≤ *γ*), then $k\left(t\right)=\sqrt{\left(t_{\max}-t\right)}/\sqrt{t_{\max}}\times \left(k_{\max}-k_{\min}\right)+k_{\min}$
 
*Rule 2*. If (*μ*_*k*_(*t*) ≤ 0.5 and *η* > *γ*), then *k*(*t*)=*τ*_1_/4+(*k*_max_+*k*_min_)/2
 
*Rule 3.* If (*μ*_*k*_(*t*) > 0.5 and *η* ≤ *γ*), then *k*(*t*)=*τ*_2_/4+*k*_min_

Here, *γ* is the threshold, and its value is 0.05; *τ*_1_ and *τ*_2_ are the parameters between [0, 1] in the rules.

On further observation of Figure 3, the purpose of *k* is to adjust the population, improve population diversity, expand the search space, and improve the global search ability of the algorithm. Therefore, the adjustment of parameter *k* based on fuzzy rules in the ROBL model can effectively improve the diversity of individual distribution in the search space. It makes up for the weak exploration ability of GWO in the late iteration. The advantage of the ROBL model over the OBL model is that the candidate solution can be obtained dynamically by parameter adjustment, which enhances the chance of the algorithm jumping out of the local optimum to a great extent. However, OBL can only obtain a fixed candidate solution. That is, parameter *k* has the ability to extend search space.

### 4.2. Equilibrium Pool Strategy

In GWO, the search is primarily guided by *α*, *β*, and *δ* wolves. If the leading wolves fall into the local optimum, the entire population will update their position in the direction of the local optimum. To address this issue, this paper introduces the equilibrium pool strategy to enhance population diversity [52]. The fundamental idea of the strategy is to calculate the fitness value of each individual after population initialization and choose three candidate solutions (***X***_1_, ***X***_2_, and ***X***_3_) based on the fitness value. Among them, ***X***_1_, ***X***_2_, and ***X***_3_ represent *α*, *β*, and *δ* wolves, respectively. In addition, the average value of three candidate solutions is calculated as the average candidate solution ***X***_*avg*_, and then the equalization pool ***X*_ ***pool* is constructed. The mathematical model is as follows:

(14) $$\begin{array}{c} \mathrm{X\_}\text{ pool}=\left(X_{1},X_{2},X_{3},X_{avg}\right),\\ X_{\mathrm{eq}}=\text{rand}\left(\mathrm{X\_}\text{ pool}\right). \end{array}$$

Here, three candidate solutions (***X***_1_, ***X***_2_, ***X***_3_) are contributed to exploitation and the average candidate solution (***X***_*avg*_) is contributed to exploration. *ω* wolf randomly selects candidate individuals from the candidate pool with equal probability for location updating. Besides, parameter ***F*** is used to balance exploration and exploitation, and the mathematical description is as follows:

(15) $$\begin{array}{c} F=\text{sign}\left(r-0.5\right)\left(e^{-\mathrm{\lambda m}}-1\right),\\ m={\left(1-t/T\right)}^{\left(t/T\right)}, \end{array}$$

where *λ* is the random vector between [0,1], *r* denotes a random number between [0,1], *sign*(*r*-0.5) is used to control the direction of exploration and exploitation, *t* represents the current number of iterations, and *T* notes the maximum number of iterations. In addition, the generation rate ***G*** is used to improve exploitation capability. The mathematical expression is as follows:

(16) $$\begin{array}{c} G=G_{0}F,\\ G_{0}=\left\{\begin{array}{cc} \text{rand}\times \left(X_{eq}-\mathrm{\lambda X}\right), & \text{rand}\geq 0.5\\ 0, & \text{rand}<0.5 \end{array}\right), \end{array}$$

where *X*_*eq*_ is a candidate solution randomly chosen from the equilibrium pool with equal probability.

In summary, when GWO applies equilibrium pool strategy, the position update formula of the individual is as follows:

(17) $$\begin{array}{c} X\left(t+1\right)=X_{eq}+\left(X\left(t\right)-X_{eq}\right)F+\frac{G}{\lambda }\left(1-F\right). \end{array}$$

### 4.3. REGWO Algorithm

It is well known that exploration and exploitation are necessary for population-based optimization algorithms, such as PSO, ABC, ACO, and so on. In standard GWO, the issue is that since all of the other individuals are attracted toward leader wolves, they may converge prematurely without enough exploration of search space, that is, standard GWO is prone to premature convergence.

To improve the performance of GWO, each grey wolf obtains the opposite solution via the ROBL strategy, which enhances individual randomness. Refraction opposite learning strategy makes up for the shortcomings of traditional opposite learning, expands the search space, and effectively enhances population diversity. In addition, an equilibrium pool strategy is introduced to reduce the likelihood of the algorithm falling into the local extremum. The equilibrium pool retains four individuals, namely *α*, *β*, and *δ* wolves as well as their mean values. The ability of exploration is properly improved by randomly selecting an individual from the equalization pool to lead the position update of *ω* wolf. The process of REGWO is described in Algorithm 1, and the flowchart of the proposed REGWO algorithm is shown in Figure 5. In REGWO, the *α*, *β*, and *δ* wolves are chosen by population initialization and fitness calculations. Then, the position is updated with equal probability by equation (3) or (17). Finally, the refraction opposite solution and its fitness value are calculated by equation (10); furthermore, the refraction solution is retained if the refraction solution is better than the original solution; otherwise, the original solution is retained. Until the end of the iteration, *α* wolf is the ultimate optimization result.

## 5. Experiments and Analysis

### 5.1. Experimental Settings

To fairly compare the performance of different algorithms, the function test set is needed. The numerical efficiency of REGWO developed in this paper was tested by solving 31 mathematical optimization problems. The first 21 benchmark functions are the classical functions utilized in literature [9, 53]; they (*f*_1_∼*f*_21_) are composed of unimodal, multimodal, fixed-dimensional multipeak, and shifted functions. The specific expressions and search intervals of these functions are shown in Table 1. The unimodal function (*f*_1_∼*f*_9_) with just one local and also global optimal solution is commonly used to evaluate the local exploitation ability of the algorithm; *f*_10_∼*f*_14_ are multimodal function and often used to test the ability of the algorithm to explore. The *f*_15_ and *f*_16_ are fixed-dimensional multipeak functions with many extreme points but low dimensions, so it is easy to optimize and can be used to assess the stability of the algorithm. The last 5 functions in Table 1 are shifted functions, which are mainly to avoid the situation that some algorithms copy one parameter to another to generate a neighbor solution [53]. The other 10 test problems (*f*_22_∼*f*_31_) considered in this paper (see Table 2) regard composite benchmark functions considered in the IEEE CEC 2019 special session [54]. These benchmark functions are more complex than the first 21 benchmark functions, and *f*_22_∼*f*_31_ are designed to have a minimum value of 1. The optimization performance of each algorithm can be further verified by solving complex problems.

Two sets of experiments are conducted in this paper. In the first experiment, REGWO is compared with some popular algorithms and novel algorithms to evaluate convergence speed and optimization accuracy. Furthermore, the comparisons of GWO, RGWOL (GWO improved only by refraction principle with linear control parameter *k*), RGWOF (GWO improved only by refraction principle with fuzzy control parameter *k*), EGWO (GWO improved only by equilibrium pool strategy), and REGWO are executed. The influences of two strategies and dynamic changes of parameter *k* on the optimization results can be observed through the experiment. In the second experiment, the comparisons of mean and standard deviation are performed between REGWO and the other six different GWO variants. Meanwhile, the population size is set to 30; the maximum number of iterations is set to 5000, and experimental results are based on 30 independent experiments.

### 5.2. Comparison with Swarm Intelligence Algorithms and Strategies Analysis

To validate the performance of the proposed REGWO algorithm in this paper, it is used to solve the functions *f*_1_∼*f*_31_, and the performance is compared with RGWOL, RGWOF, EGWO, and other swarm intelligence algorithms, including standard GWO [9], sparrow search algorithm (SSA) [55], Archimedes optimization algorithm (AOA) [56], particle swarm optimization (PSO) [57], firefly algorithm (FA) [58], and artificial bee colony (ABC) [4]. Among them, SSA and AOA are novel intelligent algorithms, and PSO, FA, and ABC are popular intelligent algorithms. For better comparison, the other parameters of algorithms are shown in Table 3.

The results on each benchmark function of the algorithms are shown in Table 4. It can be seen from Table 4 that the effectiveness of each strategy has been verified. RGWOL outperforms six test functions. RGWOF outperforms nine test functions. EGWO outperforms six test functions. Among them, the results of the RGWOF algorithm on most functions are better than RGWOL. The experimental results in Table 4 show that the effect of fuzzy control parameter *k* is better than the linear decrease of parameter *k*. Therefore, the REGWO algorithm proposed in this paper combines the equilibrium pool strategy (EGWO) with the refraction opposite learning strategy (RGWOF). At the same time, the fuzzy theory control parameter *k* is used in the refraction opposite learning. Although the RGWOF and EGWO can find the solutions, combining the two strategies has more benefits since the solutions obtained by REGWO are always better than theirs.

On the other hand, it can be seen from Table 4 that the average fitness of REGWO outperforms on 26 test functions compared with other swarm intelligence optimization algorithms. Astonishingly, REGWO can converge into the global optimal solution in solving functions *f*_1_∼*f*_3_, *f*_7_, *f*_8_, and *f*_11_∼*f*_19_, indicating that REGWO has the potential to converge to the global optimal value. On further observation in Table 4, the standard GWO is still competitive compared with SSA and AOA for unimodal functions. It is proved that the standard GWO has good exploitation ability when solving unimodal functions. However, the optimization performance of standard GWO is relatively weak for multimodal functions, while REGWO shows better performance both in unimodal functions and multimodal functions. Moreover, it can be seen from the Friedman test average rank in Table 4 that the order from low to high is REGWO, RGWOF, EGWO, RGWOL, SSA, FA, GWO, AOA, PSO, and ABC. Obviously, REGWO has preferable competitiveness compared with novel algorithms (SSA, AOA) and the classical algorithms (PSO, FA, ABC). The superior performances of REGWO should be attributed to the improved strategies. Individuals maintain high diversity during optimization due to refraction opposite solution strategy, and the equalization pool strategy weakens the leadership of the optimal solution. Therefore, the combination of the two strategies can effectively improve the performance of standard GWO in solving multimodal functions. That is to say, the ability of the algorithm to jump out of the local extremum is enhanced.

Due to the stochastic nature of these algorithms, the statistical test is necessary for providing confidential comparisons [44]. Therefore, the Wilcoxon sign rank test is conducted in this paper. The test results of the REGWO algorithm and the other 9 selected algorithms on 31 test functions are shown in Table 5. The sign + (–) denotes that the REGWO algorithm is better (worse) than its compared algorithms. The symbol = indicates that the REGWO algorithm gets the same results as its competitors. It can be seen from Table 5 that REGWO provides higher R^+^ values than R^−^ values in all cases. Moreover, the *p* values of 9 algorithms are less than 0.05, indicating that they are significantly different from REGWO, and REGWO is superior to other algorithms.

There are some reasons for REGWO has such a good performance. Firstly, the refraction principle and fuzzy control parameter are introduced in GWO; individual diversity is enhanced. RGWO improves the optimization precision and convergence speed of the standard GWO algorithm by retaining better (original solution and refraction inverse solution). Secondly, the equilibrium pool strategy enhances the global search ability of the original GWO algorithm by reducing the leadership of the leading wolves. The advantage of this strategy is particularly obvious when solving the multimodal function. Then, REGWO, as an improved GWO algorithm, combines the advantages of the two strategies. It not only improves the convergence speed of the GWO but also improves the optimization precision of the original GWO algorithm.

The convergence histories of the compared algorithms are shown in Figure 6. Through the convergence histories in Figure 6, we can find that the convergence speed of REGWO is faster than other swarm intelligence optimization algorithms on unimodal functions except *f*_5_. Although the convergence speed of the REGWO algorithm on multimodal function is not as fast as that on unimodal function, REGWO has high search precision than other algorithms. Especially, the optimization performance of REGWO is remarkable when solving more complex functions (IEEE CEC 2019 test suite). It demonstrates that REGWO algorithm not only improves the convergence speed of the standard GWO algorithm on unimodal function but also enhances the optimization precision on complex functions.

### 5.3. Comparison with GWOs

To further validate the effectiveness of the REGWO. The performances of different GWO variants are compared, and the benchmark functions (*f*_1_∼*f*_31_) are solved by REGWO, WGWO [35], DGWO [59], AGWO [60], IGWO [61], RLGWO [62], and GNHGWO [63]. To make a fair comparison, the 6 algorithms use the same parameter settings as their original literature. Then, the results are analyzed by Friedman test average rank and Wilcoxon signed-rank test, and statistical results (mean cost and standard deviation) for 30 independent experiments are reported in Table 6.

It can be seen from Table 6 that the average fitness of the REGWO is superior except for the functions *f*_5_, *f*_10_, and *f*_20_. In addition, the corresponding standard deviation is much smaller than other algorithms for most functions. The average fitness of the REGWO outperforms the other 6 enhanced GWOs on 14 benchmark functions. It can be seen that the combination of the refraction opposite learning approach and equilibrium pool strategy effectively improves the optimization accuracy of the standard GWO. The above algorithms can achieve the theoretical optimal value for the function *f*_16_. Because *f*_16_ is a fixed-dimensional multimodal function with low dimension, it is simple to solve. However, REGWO shows better stability in terms of standard deviation. The *f*_22_∼*f*_31_ are more complicated than the test functions listed in Table 1. It can better test the algorithm exploration and exploitation ability. Especially, REGWO converges to the theoretical optimal value 1 on function *f*_22_. For functions *f*_26_ and *f*_30_, the iterative optimization results of REGWO are also close to the theoretical optimal value 1. It demonstrates that REGWO still has the ability to converge to the global optimum for more complex mathematical optimization problems. Moreover, REGWO also achieves better performance in most functions in terms of standard deviation, indicating that REGWO has a better stability. From the Friedman test average rank in Table 6, the order from low to high is REGWO, IGWO, DGWO, RLGWO, AGWO, WGWO, and GNHGWO (IGWO is equal to DGWO). It shows that the performance of REGWO is much superior to other GWOs in accuracy. From the results of the Wilcoxon sign rank test in Table 7, REGWO provides higher R^+^ values than R^−^ values in all cases. Moreover, it can be seen that the *p* values of WGWO, DGWO, AGWO, IGWO, RLGWO, and GNHGWO are less than 0.05, indicating that they are significantly different from REGWO, and REGWO is far superior to the other six algorithms.

In summary, REGWO has such good performance because of the contribution of the two strategies. Firstly, the diversity of solutions is increased by refractive opposite learning. Secondly, the equilibrium pool strategy weakens the leadership of the leading wolves to increase the probability of individuals jumping out of the local optimum. Therefore, the REGWO algorithm combining two strategies is able to achieve competitive optimization results on the test problems compared with other GWOs.

## 6. Conclusion and Future Work

In order to further improve the optimization performance of GWO, this paper proposes an equalized grey wolf optimizer with refraction opposite learning (REGWO). The main idea of the algorithm is to improve the opposite learning process of OBL based on the refraction principle of light. This strategy further expands the search space of the population, increases population variety, and enhances the ability of individuals to jump out of the local extremum. At the same time, the equilibrium pool strategy is combined to weaken the leadership of the leading wolves, which effectively avoids the situation that the rest of the individuals move to the leading wolves when the leading wolves fall into the local optimum. Therefore, the combination of the two strategies effectively enhances the exploration of GWO in the late iteration. In addition, REGWO is tested on 31 benchmark functions. The experimental results show that REGWO has higher convergence speed, search accuracy, and stability compared with standard GWO, other state-of-art GWOs, and other swarm intelligence algorithms. On the whole, REGWO is more effective in solving complex optimization problem.

In our future work, the selection of search strategies still needs to be further investigated. Furthermore, the REGWO algorithm can be extended to solve multiobjective optimization, binary optimization, and application-designed problems in the future.

## Figures and Tables

**Figure 1:** Four-layer pyramid model in GWO.

**Figure 2:** 2D and 3D position vectors and the possible next position of grey wolf: (a) 2D view of grey wolf in GWO and (b) 3D view of grey wolf in GWO.

**Figure 3:** Refraction opposite learning model.

**Figure 4:** Fuzzy control structure.

**Figure 5:** The flowchart of the REGWO algorithm.

**Figure 6:** Convergence diagrams.

**Algorithm 1:** Equalized grey wolf optimizer with refraction opposite learning (REGWO).

**Table 1:** Benchmark functions (*f*_1_∼*f*_21_).

No.	Functions
*f*_1_	*f*_1_(*x*)=∑_*i*=1_^*n*^*x*_*i*_^2^
*f*_2_	*f*_2_(*x*)=∑_*i*=1_^*n*^|*x*_*i*_|+∏_*i*=1_^*n*^|*x*_*i*_|
*f*_3_	*f*_3_(*x*)=∑_*i*=1_^*n*^(∑_*i*=1_^*j*^*x*_*j*_)^2^
*f*_4_	*f*_4_(*x*)=max{|*x*_*i*_|, 1 ≤ *i* ≤ *n*}
*f*_5_	*f*_5_(*x*)=∑_*i*=1_^*n*^([*x*_*i*_+0.5])^2^
*f*_6_	*f*_6_(*x*)=∑_i=1_^n^*ix*_*i*_^4^+random[0,1)
*f*_7_	*f*_7_(*x*)=∑_*i*=1_^*n*^(10^6^)^*i* − 1/*n*−1^*x*_*i*_^2^
*f*_8_	*f*_8_(*x*)=∑_*i*=1_^*n*^*ix*_*i*_^2^
*f*_9_	*f*_9_(*x*)=∑_*i*=1_^*n*−1^[100(*x*_*i*+1_ − *x*_*i*_^2^)^2^+(*x*_*i*_ − 1)^2^]
*f*_10_	$f_{10}\left(x\right)=-20\;\exp\left(-0.2\sqrt{1/n\sum_{i=1}^{n}x_{i}^{2}}\right)-\exp\left(1/n\sum_{i=1}^{n}\cos\left(2\pi x_{i}\right)\right)+e$
*f*_11_	$f_{11}\left(x\right)=\sum_{i=1}^{n}\left[y_{i}^{2}-10\;\cos\left(2\pi y_{i}\right)+10\right],y_{i}=\left\{\begin{array}{cc} x_{i}, & \left|x_{i}\right|<0.5\\ \text{round}\left({2\text{x}}_{\text{i}}\right)/2 & \left|x_{i}\right|\geq 0.5 \end{array}\right.$
*f*_12_	$f_{12}\left(x\right)=1/4000\sum_{i=1}^{n}x_{i}^{2}-\prod_{i=1}^{n}\cos\left(x_{i}/\sqrt{i}\right)+1$
*f*_13_	*f*_13_(*x*)=1/*n*∑_*i*=1_^*n*^(*x*_*i*_^4^ − 16*x*_*i*_^2^+5*x*_*i*_)
*f*_14_	*f*_14_(*x*)=∑_*i*=1_^*n*^|*x*_*i*_ · sin(*x*_*i*_)+0.1 · *x*_*i*_|
*f*_15_	*f*_15_(*x*)=(1/500+∑_*j*=1_^25^1/∑_*i*=1_^2^(*x*_*i*_ − *a*_*ij*_)^6^)^−1^
*f*_16_	$\begin{array}{c} f_{16}\left(x\right)=\left[1+{\left(x_{1}+x_{2}+1\right)}^{2}\left(19-14x_{1}+3x_{1}^{2}-14x_{2}+6x_{1}x_{2}+3x_{2}^{2}\right)\right]*\\ \left[30+{\left(2x_{1}-3x_{2}\right)}^{2}\times \left(18-32x_{1}+12x_{1}^{2}+48x_{2}-36x_{1}x_{2}+27x_{2}^{2}\right)\right]. \end{array}$
*f*_17_	*f*_17_(*x*)=∑_*i*=1_^*n*^*z*_*i*_^2^, *z*=*x* − *o*
*f*_18_	*f*_18_(*x*)=∑_*i*=1_^*n*^(*z*_*i*_^2^ − 10 cos(2*πz*_*i*_)+10), *z*=*x* − *o*
*f*_19_	$f_{19}\left(x\right)=1/4000\sum_{i=1}^{n}z_{i}^{2}-\prod_{i=1}^{n}\cos\left(z_{i}/\sqrt{i}\right)+1,\;z=x-o$
*f*_20_	$f_{20}\left(x\right)=-20\;\exp\left(-0.2\sqrt{1/n\sum_{i=1}^{n}z_{i}^{2}}\right)-\exp\left(1/n\sum_{i=1}^{n}\cos\left(2\pi z_{i}\right)\right)+e,z=x-o$
*f*_21_	*f*_21_(*x*)=∑|*z*_*i*_ · sin(*z*_*i*_)+0.1 · *z*_*i*_|, *z*=*x* − *o*

**Table 2:** IEEE CEC 2019 test suite (*f*_22_∼*f*_31_).

No.	Function names	*F*_*i*_^*∗*^= *F*_*i*_ (*x*^*∗*^)	Dim	Range
*f*_22_ (F1)	Storn's Chebyshev polynomial fitting problem	1	9	[−8,192, 8,192]
*f*_23_ (F2)	Inverse Hilbert matrix problem	1	16	[−16,384, 16,384]
*f*_24_ (F3)	Lennard–Jones minimum energy cluster	1	18	[−4, 4]
*f*_25_ (F4)	Rastrigin's function	1	10	[−100, 100]
*f*_26_ (F5)	Griewank's function	1	10	[−100, 100]
*f*_27_ (F6)	Weierstrass function	1	10	[−100, 100]
*f*_28_ (F7)	Modified Schwefel's function	1	10	[−100, 100]
*f*_29_ (F8)	Expanded Schaffer's F6 function	1	10	[−100, 100]
*f*_30_ (F9)	Happy Cat function	1	10	[−100, 100]
*f*_31_ (F10)	Ackley function	1	10	[−100, 100]

**Table 3:** Parameter setting (PSO, FA, ABC, SSA, AOA, and GWO).

Algorithms	Parameter setting
PSO [57]	Inertia weight *w*=0.75, *b*_1_ = *b*_2_ = 2, *v*_max_=0.1^*∗*^(*x*_*max*_ − *x*_min_)
FA [58]	Light absorption coefficient *ζ* = 1, step size *s* = 0.2
ABC [4]	Control parameter *limit* = 0.6*∗*population size*∗*dim
SSA [55]	Discoverers *n* = 0.2*∗*population size
AOA [56]	Constants *d*_*1*_ = 2, *d*_*2*_ = 6, *d*_*3*_ = 1, *d*_*4*_ = 2
GWO [9]	Control parameter *a* decrease linearly from 2 to 0

**Table 4:** Search result (comparisons of PSO, FA, ABC, SSA, AOA, GWO, RGWOL, RGWOF, EGWO, and REGWO).

No.	Performance index	PSO	FA	ABC	SSA	AOA	GWO	RGWOL	RGWOF	EGWO	REGWO
*f*_1_	Mean	1.96*e*–09	1.18*e*–86	2.91*e*–11	5.22*e*–191	3.09*e*–263	1.34*e*–311	**0**	**0**	**0**	**0**
	Std	4.81*e*–09	1.90*e*–87	3.05*e*–11	0	0	0	0	0	0	0

*f*_2_	Mean	9.12*e*–02	4.56*e*–44	5.29*e*–12	1.41*e*–101	8.14*e*–165	4.26*e*–179	1.00*e*–323	**0**	3.60*e*–214	**0**
	Std	1.60*e*–01	2.49*e*–45	2.76*e*–11	7.73*e*–101	0	0	0	0	0	0

*f*_3_	Mean	6.57*e*–10	1.19*e*–44	4.88*e*+04	1.05*e*–66	7.19*e*–60	1.28*e*–75	1.13*e*–92	**0**	1.28*e*–78	**0**
	Std	1.22*e*–09	3.76*e*–44	6.73*e*+03	3.33*e*–66	2.27*e*–59	4.06*e*–75	2.11*e*–92	0	4.06*e*–78	0

*f*_4_	Mean	3.78*e*–06	1.99*e*+00	5.39*e*+01	2.21*e*–45	1.09*e*–35	1.75*e*–75	1.91*e*–241	3.32*e*–245	1.04*e*–84	**5.06*e*–251**
	Std	2.37*e*–06	2.16*e*+00	5.19*e*+00	6.99*e*–45	1.74*e*–35	4.81*e*–75	0	0	1.47*e*–84	0

*f*_5_	Mean	5.31*e*–07	**0**	3.04*e*–11	2.61*e*–32	2.99*e*–01	4.75*e*–01	6.25*e*–01	5.24*e*–01	9.05*e*–07	5.01*e*–02
	Std	1.66*e*–06	0	2.54*e*–11	3.10*e*–32	3.06*e*–01	3.43*e*–01	3.17*e*–01	2.18*e*–01	3.44*e*–07	1.05*e*–01

*f*_6_	Mean	5.32*e*–03	6.36*e*–04	2.11*e*–01	3.03*e*–04	1.02*e*–03	1.20*e*–04	7.23*e*–04	8.63*e*–05	2.74*e*–04	**2.60*e*–05**
	Std	2.93*e*–03	3.40*e*–04	4.83*e*–02	2.79*e*–04	5.02*e*–04	6.23*e*–05	5.53*e*–04	7.74*e*–05	1.37*e*–04	1.48*e*–05

*f*_7_	Mean	5.13*e*+00	5.73*e*–82	1.82*e*–09	1.76*e*–90	5.07*e*–264	6.67*e*–306	**0**	**0**	**0**	**0**
	Std	2.80*e*+01	1.30*e*–82	2.59*e*–09	9.38*e*–90	0	0	0	0	0	0

*f*_8_	Mean	1.36*e*–07	1.81*e*–87	1.17*e*–12	7.25*e*–168	1.37*e*–270	4.75*e*–312	**0**	**0**	**0**	**0**
	Std	4.32*e*–07	1.44*e*–88	9.66*e*–13	0	0	0	0	0	0	0

*f*_9_	Mean	2.87*e*+01	7.71*e*–01	3.19*e*+03	**3.12*e*–07**	2.59*e*+01	2.66*e*+01	2.71*e*+01	2.70*e*+01	2.38*e*+01	2.88*e*+00
	Std	2.09*e*+01	1.74*e*+00	1.75*e*+03	6.46*e*–07	9.00*e*–01	8.27*e*–01	1.48*e*+00	3.59*e*–02	1.30*e*+00	5.51*e*–01

*f*_10_	Mean	1.30*e*+00	2.18*e*–14	4.57*e*–05	**8.88*e*–16**	1.99*e*+01	7.99*e*–15	4.44*e*–15	4.44*e*–15	7.28*e*–15	4.44*e*–15
	Std	7.84*e*–01	5.41*e*–15	3.93*e*–05	0	1.46*e*–03	0	0	0	1.49*e*–15	0

*f*_11_	Mean	5.92*e*+01	7.33*e*+01	1.96*e*+02	**0**	1.54*e*+01	4.66*e*–01	2.53*e*–02	7.21*e*–04	2.12*e*–03	**0**
	Std	1.76*e*+01	2.21*e*+01	2.18*e*+01	0	4.19*e*+00	1.77*e*+00	3.55*e*–02	4.65*e*–03	1.42*e*–03	0

*f*_12_	Mean	2.15*e*–02	4.18*e*–03	8.41*e*–03	1.56*e*–05	1.09*e*–02	4.19*e*–04	**0**	**0**	7.39*e*–06	**0**
	Std	3.06*e*–02	7.94*e*–03	3.58*e*–02	5.77*e*–04	2.28*e*–02	2.29*e*–03	0	0	2.32*e*–05	0

*f*_13_	Mean	−6.65*e*+01	−7.08*e*+01	−5.13*e*+01	−7.20*e*+01	−6.93*e*+01	−6.31*e*+01	−7.58*e*+01	−7.62*e*+01	−6.80*e*+01	**−7.83*e*+01**
	Std	2.76*e*+00	2.28*e*+00	1.79*e*+00	2.36*e*+00	2.83*e*+00	3.36*e*+00	3.82*e*–13	1.62*e*–13	2.23*e*+00	2.34*e*–14

*f*_14_	Mean	4.84*e*–03	6.31*e*–15	2.26*e*+01	1.54*e*–17	2.89*e*–04	2.81*e*–170	1.37*e*–319	1.33*e*–322	8.72*e*–13	**0**
	Std	4.02*e*–03	3.27*e*–15	1.89*e*+00	2.53*e*–17	3.79*e*–04	0	0	0	2.75*e*–12	0

*f*_15_	Mean	3.55*e*+00	1.06*e*+00	1.39*e*+00	6.51*e*+00	9.97*e*–01	4.26*e*+00	1.65*e*+00	6.21*e*+00	**9.98*e*–01**	**9.98*e*–01**
	Std	3.16*e*+00	3.62*e*–01	1.81*e*+00	5.76*e*+00	1.63*e*–06	4.23*e*+00	1.14*e*+00	5.59*e*+00	6.25*e*–13	1.82*e*–12

*f*_16_	Mean	**3.00*e*+00**	**3.00*e*+00**	**3.00*e*+00**	**3.00*e*+00**	**3.00*e*+00**	**3.00*e*+00**	**3.00*e*+00**	**3.00*e*+00**	**3.00*e*+00**	**3.00*e*+00**
	Std	1.09*e*–15	1.22*e*–15	2.71*e*–07	9.70*e*–16	1.50*e*–07	2.66*e*–07	3.15*e*–07	3.73*e*–07	7.40*e*–16	4.44*e*–16

*f*_17_	Mean	4.54*e*–10	1.20*e*–86	1.42*e*–10	4.30*e*–192	9.24*e*–269	1.15*e*–310	**0**	**0**	**0**	**0**
	Std	1.40*e*–09	2.11*e*–87	3.86*e*–10	0	0	0	0	0	0	0

*f*_18_	Mean	5.23*e*+01	6.31*e*+01	2.12*e*+02	6.61*e*–04	1.42*e*+01	7.61*e*–02	3.51*e*–08	2.89*e*–10	3.51*e*–10	**0**
	Std	1.49*e*+01	2.01*e*+01	1.03*e*+01	4.97*e*–03	7.59*e*+00	4.97*e*–01	2.28*e*–07	1.53*e*–09	9.52*e*–09	0

*f*_19_	Mean	3.61*e*–02	1.72*e*–03	5.27*e*–04	3.17*e*–06	2.10*e*–03	2.17*e*–04	8.27*e*–108	**0**	1.72*e*–03	**0**
	Std	2.93*e*–02	4.21*e*–03	4.80*e*–04	1.66*e*–06	6.67*e*–03	1.66*e*–04	0	0	5.44*e*–03	0

*f*_20_	Mean	2.04*e*+00	2.57*e*–14	5.54*e*–05	**8.88*e*–16**	1.99*e*+01	7.99*e*–15	4.44*e*–12	4.44*e*–15	7.63*e*–15	4.44*e*–15
	Std	7.38*e*–01	8.53*e*–15	4.13*e*–05	0	1.93*e*–03	0	0	0	1.12*e*–15	0
*f*_21_	Mean	8.50*e*–11	5.26*e*–16	2.22*e*–02	9.54*e*–18	4.86*e*–03	5.87*e*–05	5.56*e*–11	2.62*e*–13	3.12*e*–08	**1.54*e*–46**
	Std	1.43*e*–10	4.41*e*–15	2.39*e*–01	1.79*e*–17	2.21*e*–02	2.28*e*–04	9.24*e*–10	7.55*e*–12	1.56*e*–07	8.43*e*–46

*f*_22_	Mean	2.01*e*+04	2.55*e*+03	7.02*e*+06	**1.00*e*+00**	3.63*e*+02	4.77*e*+03	1.50*e*+00	1.21*e*+00	1.18*e*+03	**1.00*e*+00**
	Std	2.98*e*+04	4.41*e*+03	2.62*e*+06	0	9.35*e*+02	1.39*e*+04	7.65*e*–15	0	2.72*e*+03	0

*f*_23_	Mean	2.48*e*+02	3.75*e*+02	7.63*e*+03	4.25*e*+01	1.99*e*+02	1.57*e*+02	6.27*e*+00	5.23*e*+00	7.59*e*+01	**4.26*e*+00**
	Std	1.22*e*+02	1.40*e*+02	1.13*e*+03	2.60*e*–01	1.29*e*+02	1.08*e*+02	4.79*e*–02	2.73*e*–02	5.39*e*+01	3.85*e*–02

*f*_24_	Mean	4.36*e*+00	5.52*e*+00	1.20*e*+01	7.43*e*+00	2.95*e*+00	5.21*e*+00	4.59*e*+00	5.02*e*+00	4.42*e*+00	**2.04*e*+00**
	Std	3.13*e*+00	2.83*e*+00	4.12*e*–01	2.65*e*+00	1.86*e*+00	3.20*e*+00	1.08*e*+00	6.63*e*–01	2.67*e*+00	1.11*e*–00

*f*_25_	Mean	2.52*e*+01	1.43*e*+01	2.72*e*+01	3.80*e*+01	3.02*e*+01	1.37*e*+01	1.45*e*+01	1.01*e*+01	7.76*e*+00	**5.87*e*+00**
	Std	1.09*e*+01	5.83*e*+00	3.62*e*+00	1.18*e*+01	7.47*e*+00	6.43*e*+00	8.07*e*+00	7.02*e*+00	2.60*e*+00	3.49*e*+00

*f*_26_	Mean	1.14*e*+00	**1.06*e*+00**	1.29*e*+00	1.23*e*+00	1.83*e*+00	1.94*e*+00	1.62*e*+00	1.48*e*+00	1.19*e*+00	1.16*e*+00
	Std	4.71*e*–02	2.95*e*–02	3.47*e*–02	1.63*e*–01	2.20*e*–01	1.12*e*+00	1.98*e*–01	2.39*e*–01	6.74*e*–02	6.89*e*–02

*f*_27_	Mean	2.83*e*+00	1.63*e*+00	9.18*e*+00	5.46*e*+00	3.53*e*+00	2.69*e*+00	2.61*e*+00	2.28*e*+00	2.26*e*+00	**1.56*e*+00**
	Std	1.38*e*+00	8.87*e*–01	7.59*e*–01	1.43*e*+00	1.85*e*+00	1.03*e*+00	6.85*e*–01	1.06*e*+00	1.33*e*+00	1.08*e*+00

*f*_28_	Mean	8.45*e*+02	4.63*e*+02	1.48*e*+03	8.96*e*+02	5.42*e*+02	7.62*e*+02	5.31*e*+02	7.39*e*+02	2.75*e*+02	**2.16*e*+02**
	Std	2.72*e*+02	2.75*e*+02	1.70*e*+02	2.50*e*+02	2.09*e*+02	3.17*e*+02	3.59*e*+02	3.22*e*+02	1.72*e*+02	1.35*e*+02

*f*_29_	Mean	4.06*e*+00	3.84*e*+00	5.07*e*+00	4.28*e*+00	3.47*e*+00	3.78*e*+00	3.77*e*+00	3.22*e*+00	3.25*e*+00	**2.96*e*+00**
	Std	4.90*e*–01	2.96*e*–01	7.67*e*–02	4.13*e*–01	6.17*e*–01	5.17*e*–01	3.27*e*–01	4.09*e*–01	5.21*e*–01	6.79*e*–01

*f*_30_	Mean	1.14*e*+00	1.08*e*+00	1.18*e*+00	1.38*e*+00	1.19*e*+00	1.09*e*+00	1.11*e*+00	1.19*e*+00	1.10*e*+00	**1.04*e*+00**
	Std	3.76*e*+00	2.11*e*–02	2.31*e*–02	2.06*e*–01	1.09*e*–01	6.76*e*–02	6.13*e*–02	6.87*e*–02	2.63*e*–02	2.96*e*–02

*f*_31_	Mean	2.09*e*+01	1.31*e*+01	2.12*e*+01	2.10*e*+01	2.11*e*+01	2.05*e*+01	1.88*e*+01	1.87*e*+01	1.94*e*+01	**1.12*e*+01**
	Std	2.88*e*–03	1.04*e*+01	7.46*e*–02	8.72*e*–02	1.37*e*–01	2.40*e*+00	5.28*e*+00	1.17*e*–01	6.06*e*+00	1.05*e*+01

Friedman test average rank		**7.85**	**5.83**	**8.69**	**5.59**	**6.83**	**5.91**	**4.50**	**3.67**	**4.17**	**1.90**

**Table 5:** Results of Wilcoxon signed-rank test (comparison with PSO, FA, ABC, SSA, AOA, GWO, RGWOL, RGWOF, and EGWO).

Case	+/=/−	*R*−	*R* ^+^	*p* value
REGWO vs. PSO	30/1/0	21	444	1.36*e*–05
REGWO vs. FA	28/1/2	55	410	2.61*e*–04
REGWO vs. ABC	30/1/0	11	454	5.21*e*–06
REGWO vs. SSA	25/3/3	57	349	8.85*e*–04
REGWO vs. AOA	30/1/0	10	455	4.72*e*–06
REGWO vs. GWO	30/1/0	0	465	1.73*e*–06
REGWO vs. RGWOL	24/7/0	123	276	2.70*e*–05
REGWO vs. RGWOF	20/11/0	178	210	8.85*e*–05
REGWO vs. EGWO	25/6/0	96	311	6.45*e*–05

**Table 6:** Search result comparisons of GWOs.

No.	Performance index	WGWO	DGWO	AGWO	IGWO	RLGWO	GNHGWO	REGWO
*f*_1_	Mean	**0**	**0**	**0**	3.72*e*–317	**0**	1.02*e*–04	**0**
	Std	0	0	0	0	0	2.18*e*–04	0

*f*_2_	Mean	2.41*e*–200	**0**	1.82*e*–281	1.69*e*–187	**0**	1.64*e*–04	**0**
	Std	0	0	0	0	0	2.93*e*–04	0

*f*_3_	Mean	8.92*e*–98	1.80*e*–172	1.46*e*–144	1.53*e*–62	**0**	2.09*e*–03	**0**
	Std	2.82*e*–97	0	4.64*e*–144	4.53*e*–62	0	1.14*e*–03	0

*f*_4_	Mean	5.31*e*–82	3.54*e*–151	3.00*e*–128	7.94*e*–60	3.54*e*–46	5.59*e*–03	**3.06*e*–252**
	Std	2.28*e*–81	1.11*e*–150	1.64*e*–128	3.25*e*–59	1.84*e*–45	1.83*e*–02	0

*f*_5_	Mean	5.90*e*–01	5.56*e*–01	1.03*e*+00	**1.09*e*–27**	4.75*e*–01	6.85*e*+00	1.66*e*–02
	Std	2.94*e*–01	3.55*e*–01	4.55*e*–01	9.26*e*–27	2.48*e*–01	3.08*e*–01	6.35*e*–02

*f*_6_	Mean	1.53*e*–04	2.14*e*–04	3.59*e*–05	6.72*e*–04	8.89*e*–04	1.28*e*–05	**7.43*e*–06**
	Std	6.91*e*–04	1.14*e*–04	5.84*e*–05	9.98*e*–04	9.56*e*–04	1.61*e*–05	1.38*e*–06

*f*_7_	Mean	**0**	**0**	**0**	**0**	**0**	3.52*e*–03	**0**
	Std	0	0	0	0	0	1.72*e*–02	0

*f*_8_	Mean	**0**	**0**	**0**	**0**	**0**	3.15*e*–08	**0**
	Std	0	0	0	0	0	1.02*e*–07	0

*f*_9_	Mean	5.68*e*+00	6.51*e*+00	6.00*e*+00	5.75*e*+00	6.75*e*+00	8.83*e*+00	**2.99*e*+00**
	Std	7.70*E*–01	6.68*e*–01	3.93*e*–01	4.23*e*+00	1.02*e*+00	3.51*e*–01	5.53*e*–01

*f*_10_	Mean	7.51*e*–15	7.99*e*–15	6.21*e*–15	7.63*e*–15	**1.24*e*–15**	1.73*e*–03	4.44*e*–15
	Std	1.22*e*–15	0	1.77*e*–15	1.08*e*–15	1.12*e*–15	3.36*e*–03	0

*f*_11_	Mean	**0**	**0**	**0**	3.70*e*+00	**0**	8.65*e*–06	**0**
	Std	0	0	0	1.82*e*+00	0	2.73*e*–05	0

*f*_12_	Mean	**0**	8.20*e*–03	**0**	1.45*e*–02	**0**	6.51*e*–07	**0**
	Std	0	1.17*e*–02	0	1.39*e*–02	0	1.25*e*–06	0

*f*_13_	Mean	−7.22*e*+01	−7.25*e*+01	−7.46*e*+01	−7.74*e*+01	−7.23*e*+01	−5.82*e*+01	**−7.83*e*+01**
	Std	3.43*e*+00	4.01*e*+00	2.80*e*+00	1.31*e*+00	3.80*e*+00	3.74*e*+00	1.25*e*+00

*f*_14_	Mean	**0**	**0**	**0**	1.42*e*–07	4.63*e*–06	2.60*e*–07	**0**
	Std	0	0	0	4.51*e*–07	1.15*e*–05	5.86*e*–07	0

*f*_15_	Mean	1.39*e*+00	4.53*e*+00	3.54*e*+00	**9.98*e*–01**	4.90*e*+00	1.06*e*+00	**9.98*e*–01**
	Std	8.36*e*–01	4.39*e*+00	3.91*e*+00	5.03*e*–01	5.02*e*+00	1.44*e*–01	1.81*e*–12

*f*_16_	Mean	**3.00*e*+00**	**3.00*e*+00**	**3.00*e*+00**	**3.00*e*+00**	**3.00*e*+00**	**3.00*e*+00**	**3.00*e*+00**
	Std	3.63*e*–07	5.57*e*–07	3.33*e*–07	2.17*e*–15	3.89*e*–07	1.94*e*–02	1.18*e*–15

*f*_17_	Mean	**0**	**0**	**0**	**0**	**0**	4.66*e*–06	**0**
	Std	0	0	0	0	0	1.43*e*–05	0

*f*_18_	Mean	**0**	**0**	**0**	3.97*e*–01	**0**	3.83*e*–10	**0**
	Std	0	0	0	1.20*e*–01	0	8.87*e*–10	0

*f*_19_	Mean	7.44*e*–04	2.35*e*–03	**0**	2.02*e*–02	6.26*e*–06	5.09*e*–06	**0**
	Std	2.46*e*–03	3.61*e*–03	0	2.49*e*–02	4.12*e*–05	1.59*e*–05	0

*f*_20_	Mean	4.44*e*–15	4.41*e*–15	4.44*e*–15	4.43*e*–15	**8.88*e*–16**	7.16*e*–07	4.44*e*–15
	Std	0	0	9.01*e*–16	0	1.70*e*–15	1.16*e*–04	0

*f*_21_	Mean	1.77*e*–07	2.44*e*–06	9.87*e*–09	5.01*e*–14	6.54*e*–10	4.14*e*–06	**1.54*e*–46**
	Std	6.75*e*–07	1.26*e*–05	5.40*e*–08	2.58*e*–13	5.88*e*–09	6.09*e*–06	8.43*e*–46

*f*_22_	Mean	2.85*e*+01	1.98*e*+04	8.64*e*+01	1.29*e*+03	**1.00*e*+00**	**1.00*e*+00**	**1.00*e*+00**
	Std	5.43*e*+01	6.25*e*+04	2.48*e*+02	1.90*e*+03	0	6.83*e*–06	6.37*e*–15

*f*_23_	Mean	4.68*e*+00	4.62*e*+00	4.64*e*+00	4.31*e*+00	4.89*e*+00	4.98*e*+00	**4.24*e*+00**
	Std	3.53*e*–01	3.73*e*–01	3.98*e*–01	2.77*e*–01	2.61*e*–01	8.71*e*–02	4.77*e*–02

*f*_24_	Mean	4.75*e*+00	3.27*e*+00	5.39*e*+00	7.19*e*+00	4.83*e*+00	9.07*e*+00	**1.46*e*+00**
	Std	3.01*e*+00	3.06*e*+00	3.54*e*+00	1.69*e*+00	3.28*e*+00	8.73*e*–01	4.87*e*–00

*f*_25_	Mean	1.33*e*+01	1.64*e*+01	1.65*e*+01	8.19*e*+00	2.01*e*+01	7.50*e*+01	**7.64*e*+00**
	Std	5.30*e*+00	8.47*e*+00	8.05*e*+00	2.09*e*+00	6.01*e*+00	9.40*e*+00	1.14*e*+00

*f*_26_	Mean	1.39*e*+00	1.42*e*+00	1.63*e*+00	1.42*e*+00	1.42*e*+01	4.74*e*+01	**1.16*e*+00**
	Std	2.30*e*–01	2.41*e*–01	7.57*e*–01	6.68*e*–02	3.91*e*+01	8.78*e*+00	8.47*e*–02

*f*_27_	Mean	2.46*e*+00	2.17*e*+00	3.88*e*+00	1.51*e*+00	2.77*e*+00	1.00*e*+01	**1.50*e*+00**
	Std	8.17*e*–01	9.82*e*–01	3.57*e*–01	1.24*e*+00	1.65*e*+00	7.06*e*–01	6.23*e*–01

*f*_28_	Mean	5.54*e*+02	6.64*e*+02	6.04*e*+02	2.82*e*+02	7.79*e*+02	1.60*e*+03	**2.17*e*+02**
	Std	2.41*e*+02	2.91*e*+02	2.37*e*+02	2.70*e*+02	3.37*e*+02	1.49*e*+02	2.19*e*+02

*f*_29_	Mean	3.72*e*+00	3.73*e*+00	4.02*e*+00	3.18*e*+00	3.69*e*+00	4.96*e*+00	**2.69*e*+00**
	Std	6.63*e*–01	6.74*e*–01	4.03*e*–01	6.61*e*–01	4.71*e*–01	1.47*e*–01	7.66*e*–01

*f*_30_	Mean	1.11*e*+00	1.10*e*+00	1.14*e*+00	1.09*e*+00	1.13*e*+00	2.80*e*+00	**1.06*e*+00**
	Std	5.04*e*–02	5.58*e*–02	3.89*e*–02	3.48*e*–02	6.24*e*–02	5.32*e*–01	2.88*e*–02

*f*_31_	Mean	2.13*e*+01	2.13*e*+01	2.07*e*+01	1.99*e*+01	2.10*e*+01	2.13*e*+01	**1.11*e*+01**
	Std	9.81*e*–02	1.98*e*+00	9.55*e*–02	6.42*e*+00	1.38*e*–01	9.34*e*–02	9.80*e*+00
Friedman test average rank		**3.85**	**3.98**	**4.09**	**3.98**	**4.04**	**6.09**	**1.93**

**Table 7:** Results of Wilcoxon signed-rank test (comparison with GWOs).

Case	+/ = /−	*R*−	*R* ^+^	*p* value
REGWO vs. WGWO	21/10/0	127	231	5.95*e*–05
REGWO vs. DGWO	22/9/0	117	250	6.08*e*–05
REGWO vs. AGWO	20/11/0	146	210	8.85*e*–05
REGWO vs. IGWO	25/5/1	72	334	5.68*e*–05
REGWO vs. RLGWO	20/9/2	161	205	1.89*e*–04
REGWO vs. GNHGWO	29/2/0	21	435	2.56*e*–06

## Data Availability

The data used to support the findings of this study are available from the corresponding author upon request.
